# Development and Validation of Deep Learning Models for the Multiclassification of Reflux Esophagitis Based on the Los Angeles Classification

**DOI:** 10.1155/2023/7023731

**Published:** 2023-02-18

**Authors:** Hailong Ge, Xin Zhou, Yu Wang, Jian Xu, Feng Mo, Chen Chao, Jinzhou Zhu, Weixin Yu

**Affiliations:** ^1^Department of General Surgery, Jintan Affiliated Hospital of Jiangsu University, Changzhou 213200, China; ^2^Department of Gastroenterology, Jintan Affiliated Hospital of Jiangsu University, Changzhou 213200, China; ^3^Department of Gastroenterology, The First Affiliated Hospital of Soochow University, Suzhou 215000, China

## Abstract

This study is to evaluate the feasibility of deep learning (DL) models in the multiclassification of reflux esophagitis (RE) endoscopic images, according to the Los Angeles (LA) classification for the first time. The images were divided into three groups, namely, normal, LA classification A + B, and LA C + D. The images from the HyperKvasir dataset and Suzhou hospital were divided into the training and validation datasets as a ratio of 4 : 1, while the images from Jintan hospital were the independent test set. The CNNs- or Transformer-architectures models (MobileNet, ResNet, Xception, EfficientNet, ViT, and ConvMixer) were transfer learning via Keras. The visualization of the models was proposed using Gradient-weighted Class Activation Mapping (Grad-CAM). Both in the validation set and the test set, the EfficientNet model showed the best performance as follows: accuracy (0.962 and 0.957), recall for LA A + B (0.970 and 0.925) and LA C + D (0.922 and 0.930), Marco-recall (0.946 and 0.928), Matthew's correlation coefficient (0.936 and 0.884), and Cohen's kappa (0.910 and 0.850), which was better than the other models and the endoscopists. According to the EfficientNet model, the Grad-CAM was plotted and highlighted the target lesions on the original images. This study developed a series of DL-based computer vision models with the interpretable Grad-CAM to evaluate the feasibility in the multiclassification of RE endoscopic images. It firstly suggests that DL-based classifiers show promise in the endoscopic diagnosis of esophagitis.

## 1. Introduction

Gastroesophageal reflux disease (GERD) is a condition in which gastroesophageal reflux leads to esophageal mucosal lesions and troublesome symptoms [1, 2]. It is classified into reflux esophagitis (RE) with mucosal injuries and nonerosive reflux disease (NERD) only with symptoms [3]. Recently, the prevalence of RE has increased in Eastern Asia, due to the westernized lifestyle and diet [4, 5]. The severe complications of RE include ulcer bleeding and strictures. Even though RE-induced death is rare, these severe complications are related with significant morbidity and mortality rates [6].

According the Japan's 3^rd^ guideline [3] and the Lyon Consensus [1], the paradigm of GERD diagnosis hinges on the identification of esophageal mucosal lesions and then the grading of the severity of esophagitis. In general, GERD is generally evaluated by clinical symptoms or responses to antisecretory therapy; however, the diagnosis required endoscopy and reflux monitoring [7]. Endoscopy is necessary to the grading of esophagitis, which plays a key role in the algorithms for the diagnosis and treatment of GERD [3]. The Los Angeles (LA) classification is the most widely used and validated scoring system to describe the endoscopic appearance of esophageal mucosa and stratify its severity [8].

Deep learning (DL) is a statistical learning method that empowers computers to extract features of raw data, including structured data, images, text, and audio, without human intervention. The remarkable progress of DL-based artificial intelligence (AI) has reshaped various aspects of clinical practice [9]. DL presents a significant advantage in the fields of computer vision to analyze medical images and videos containing gigantic quantities of information [10]. In gastroenterology, AI is increasingly being integrated into computer-aided diagnosis (CAD) systems to improve lesions detection and characterization in endoscopy [11]. To our best knowledge, there were no previous reports concerning the application of DL in the endoscopic classification of RE.

In this multicentral retrospective study, we aimed to evaluate the feasibility of DL models in the multiclassification of RE endoscopic images, according to the LA classification.

## 2. Methods

### 2.1. Datasets

Subjects who underwent the upper endoscopy were recruited from two hospitals as follows: (1) Suzhou: The First Affiliated Hospital of Soochow University and (2) Jintan: Affiliated Hospital of Jiangsu University, between 2015 and 2021. In the two centers, subjects were excluded if they have (1) esophagitis of other etiologies, e.g., pills-induced esophagitis, eosinophilic, radiation, and infectious esophagitis; (2) esophageal varices; (3) esophageal squamous cell cancer. This study was approved by the Ethics Committee of The First Affiliated Hospital of Soochow University and conducted in accordance with the Helsinki Declaration of 1975 as revised in 2000 (the IRB approval number 2022098). All participants signed statements of informed consent before inclusion. Besides, the Z-line endoscopic images were also obtained from an open dataset, HyperKvasir, which now is the largest dataset of the gastrointestinal endoscopy (https://datasets.simula.no/hyper-kvasir/) [12]. The dataset offers labeled/unlabeled/segmented image data and annotated video data from Bærum Hospital in Norway. The characteristic of the datasets was shown in Figure 1. Each endoscopic image of Z-line was determined and labeled as normal, LA classification A + B (LA A + B), or LA classification C + D (LA C + D) by three rich-experienced endoscopists, based on the LA classification. The endoscopic devices in our hospital include Olympus GIF-Q260, GIF-H290, and Fuji EG-601WR, while in the HyperKvasir dataset, they include Olympus and Pentax at the Department of Gastroenterology, Bærum Hospital.

### 2.2. Models

#### 2.2.1. CNNs-Based Architectures

Pretrained convolutional neural networks (CNNs) include convolutional layers, average pooling layers, and fully connected layers, with ReLU activation. Besides, two dense layers (ReLU activation) and one dense layer (Softmax activation) were added on the top of the pretrained CNNs layers for feature extraction, as shown in Figure 2(a).

#### 2.2.2. Transformer-Based Architectures

Transformer is characterized by synchronous input based on the self-attention mechanism. The Transformer encoder consists of three main components, namely, input embedding, multihead attention, and feed-forward neural networks. Similar as the CNNs, following them, three dense layers (ReLU or Softmax activation) were added on the top of the pretrained Transformer-based architectures.

#### 2.2.3. Pretrained Models

The six CNNs-or Transformer-architectures models, i.e., MobileNet (MobileNet V1), ResNet (ResNet50 V2), Xception (Xception V1), EfficientNet (EfficientNet V2 small), ViT (ViT B/16), and ConvMixer (ConvMixer-768/32) were selected. These computer vision models were previously trained on the ImageNet database (https://www.image-net.org). The pretrained models and parameters were obtained from Keras or TensorFlow Hub (https://hub.tensorflow.google.cn/).

### 2.3. Training and Validation

#### 2.3.1. Implementation

The CNNs-or Transformer-architectures models were transfer learning via Keras (TensorFlow framework as backbone). The Adam optimizer and the categorical cross-entropy cost function, with a fixed learning rate of 0.0001 and a batch size of 32, were compiled in the training of models. A link to the codes concerning the training procedure could be obtained here on https://osf.io/4tdhu/?view_only=b279429b6a284ad885da7cad79126df7.

#### 2.3.2. Target Training

Endoscopic images of Z-line were saved as JPEG format. All images were rescaled to 331 × 331 pixels and then the pixel values were normalized from 0 to 255 to 0 to 1. Based on the LA classification, the images were divided into three groups, namely, normal, LA A + B, and LA C + D. Images from the HyperKvasir dataset and Suzhou hospital were divided into the training and validation datasets as a ratio of 4 : 1. The flowchart of the study was plotted in Figure 2(b).

#### 2.3.3. External Test

A total of 600 endoscopic images (as JPEG format) from Jintan hospital were the external test set, including 300 normal, 200 LA A + B, and 100 LA C + D (Figure 2(b)). The endoscopic devices in Jintan hospital include Olympus GIF-Q260 and GIF-H290.

#### 2.3.4. Comparison with Endoscopists

To further evaluate the performance of the models, the images from the test dataset were determined by two endoscopists (junior, five-year endoscopic experience, and senior, more than ten-year experience).

#### 2.3.5. Visualization of the Model

The visualization of the models was proposed using Gradient-weighted Class Activation Mapping (Grad-CAM) [13]. Grad-CAM uses the class-specific gradient information into the final convolutional layers of CNNs-based architectures to create projecting maps of the key areas in the images without retraining. Based on the best multiclassification model, the Grad-CAM technology was to offer inferential explanation on the original images.

### 2.4. Statistical Analysis

The training of the models was performed on Python (version: 3.9) and TensorFlow (2.8.0). The performance was mainly evaluated by accuracy and recall. True positives (TP), true negatives (TF), false positives (FP), and false negatives (FN) were enumerated to assess the classifiers. Formulas were as follows: Accuracy = (TP + TN)/(TP + FP + FN + TN), recall = TP/(TP + FN), Marco-recall = mean recalls, Matthew's correlation coefficient (MCC) = (TP *∗* TN − FP *∗* FN)/√(TP + FP) (TP + FN) (TN + FP) (TN + FN), and Cohen's kappa *k* = (p0 − pe)/(1 − pe) (p0: relative observed agreement among raters; pe: hypothetical probability of chance agreement).

## 3. Results

### 3.1. Performance in the Validation Set

The confusion matrix of the six models in the validation set was plotted in Figure 3(a). The EfficientNet model showed the highest accuracy of 0.962, followed by the ConvMixer model (0.950) and Xception (0.938) (Table 1). The recalls for LA A + B and LA C + D of the EfficientNet model were 0.970 and 0.922, while its Marco-recall was 0.946. In term of multiclass metrics, its MCC and Cohen's kappa were also highest (0.936 and 0.910).

### 3.2. Performance in the Test Set

The confusion matrix in the test set was plotted in Figure 3(b)). The EfficientNet model still presented the best performance. Its accuracy was 0.957, followed by ConvMixer (0.943) and Xception (0.936) (Table 1). Moreover, the recalls for LA A + B and LA C + D of the EfficientNet model were 0.925 and 0.930, while its Marco-recall reached 0.928, better than the other models. In term of multiclass metrics, its MCC and Cohen's kappa were still highest (0.884 and 0.850).

### 3.3. Comparison with the Endoscopists

In the test set, the junior endoscopist presented an accuracy of 0.916, recalls for LA A + B 0.885 and LA C + D 0.840, Marco-recall 0.863, MCC 0.820, and Cohen's kappa 0.780 (Table 1). In the meantime, the senior endoscopist showed an accuracy of 0.945, recalls for LA A + B 0.905 and LA C + D 0.890, Marco-recall 0.898, MCC 0.864, and Cohen's kappa 0.830.

### 3.4. The Grad-CAM Heatmap

According to the gradient information of the last convolution layer of the EfficientNet model, the Grad-CAM was plotted and highlighted the lesions of the original images (Figure 4). The left column displays the original endoscopic images. The middle column illustrates the Grad-CAM heatmap on the output of the last convolution layer. The right column shows the Grad-CAM heatmap added to the original endoscopic images, in which the highlighted regions reflect the lesions determined by the EfficientNet model.

The left column displays the original endoscopic images. The middle column illustrates the Grad-CAM heatmap on the output of the last convolution layer. The right column shows the Grad-CAM heatmap added to the original endoscopic images, in which the highlighted regions reflect the lesions determined by the EfficientNet model.

## 4. Discussion

This study proposed a series of multiclassification computer vision models with the interpretable Grad-CAM to evaluate the feasibility of DL in the endoscopic images of RE, according to the LA classification. Six CNNs-or Transformer-architectures models were developed and the EfficientNet model showed practicable performance, better than the endoscopists.

In 1999, Lundell et al. [8] developed the LA classification to describe the mucosal appearance in endoscopy and to assess its correlation with the clinical changes in patients with RE. It was developed for the purpose of stratifying clinically relevant severity of RE. According to the LA classification, type A is defined as one (or more) mucosal break, no longer than 5 mm-long, that does not extend between the tops of two mucosal folds; type B is defined as one (or more) mucosal break, more than 5 mm, that still does not extend between the tops of two folds; type C is defined as one (or more) mucosal break that is continuous between the tops of two or more mucosal folds but which is no longer than 3/4 of the esophageal circumference; type D is defined as one (or more) mucosal break that is more than 3/4 of the circumference [8]. According to the Japan 2021 guideline [3] and the ACG 2021 guideline [7], RE is classified into mild RE (grade A or B of LA classification) and severe RE (grade C or D), in which the latter was defined as the high grade of RE, based on the Lyon Consensus [1]. The stratification is essential to the detailed diagnosis and the decision-making of therapy [3]. Thus, in this study, we labeled the images and trained the multiclassification models based on the forementioned guidelines. AI is being widely applied in a variety of clinical settings aiming to improve the management of the gastrointestinal diseases [14]. DL is a subset of machine learning that can automatically extract features of input data via artificial neural networks, organized as CNNs and Transformer [15]. The past five years witness a series of studies assessing the performance of DL in the diagnosis of esophageal diseases [16–22]. The main application is the computer vision task, consisting of the detection and segmentation lesions in esophageal endoscopic images or video [23, 24]. The CAD system is designed to detect and differentiate lesions based on the mucosal/vascular pattern, to stratify the progression of the diseases or to assist the decision-making of therapy [20, 25, 26]. The remarkable advantage is reducing the workload of endoscopists and improving diagnostic accuracy [27, 28].

Recently, Visaggi et al. [29] performed a meta-analysis concerned machine learning in the diagnosis of esophageal diseases. According to their review, there were a total of 42 studies. Among them, nine were focused on Barrett's esophagus and three were about GERD [30–32]. In terms of DL, Ebigbo et al. [33] developed a real-time endoscopic system to classify normal Barrett's esophagus and early esophageal adenocarcinoma, which showed an accuracy of 89.9%. Similarly, a CAD system by de Groof et al. [19] was used to improve the detection of dysplastic Barrett's esophagus. The ResNet/UNet-based system showed the performance of high accuracy detection and near-perfect segmentation, better than general endoscopists. One month ago, Tang et al. [17] trained a multitask DL model to diagnose esophageal lesions (normal vs. cancer vs. esophagitis). According to their report, the model achieved a high accuracy (93.43%) in complex classification, as well as a satisfied coefficient (77.84%) in semantic segmentation. Guimaraes et al. [18] proposed a CNNs-based multiclassification model (normal vs. eosinophilic esophagitis vs. candidiasis). In the test set, the model presented a fine global accuracy (0.915), higher than endoscopists.

In this multicentral study, six CNNs-or Transformer-architectures computer vision models were transfer learning to the multiclassification of RE endoscopic images, according to the LA classification. The EfficientNet model displayed the highest accuracy and Marco-recall. EfficientNet is a CNNs architecture and scaling method that uniformly scales all dimensions with a set of fixed scaling coefficients [34]. There are various models designed to improve training efficiency, e.g., Transformer blocks in Transformers-architectures models. But expensive overhead depending on parameter size comes as an issue. EfficientNetV2 is the successor of EfficientNet, which is a family of models optimized for floating point operations and parameter efficiency. In 2021, Google used a combination of training-aware neural architecture search, scaling to further optimize the training speed and parameter efficiency to develop this new family [35]. EfficientNetV2 overcomes some of the training bottlenecks and outperforms the V1 models. Moreover, compared with Transformer-architectures models, EfficientNet shows advantage in this small dataset with limited computing power. In the comparison with the endoscopists, the EfficientNet model also showed advantages both in accuracy and recall. Interpretability for a DL model has been one of the essential respects. Computer scientists and medical practitioners are showing more concerns about the inference of AI during the development of models, especially in the field of computer vision. Therefore, lastly, we proposed the Grad-CAM technology to visualize the inferential explanation on the original images.

Our study has some limitations. To begin with, we only focus on esophagitis caused by reflex, rather than various etiologies, e.g., radiation, eosinophilic, and pill-induced esophagitis. Further studies, based on medical history and biopsy, are required to develop more complex classifiers for esophagitis. Besides, the images dataset was limited, while video files were not involved in the analyzation. This study still required more data for validation. Lastly, we did not deploy the models in endoscopic devices. We believe that this study may contribute to the future deployment in the actual practice.

## 5. Conclusions

In this study, we developed a series of DL-based computer vision models with the interpretable Grad-CAM to evaluate the feasibility of AI in the multiclassification of RE endoscopic images for the first time. It suggests that DL-based classifiers show promise in the endoscopic diagnosis of esophagitis. In the future, it is necessary to investigate the multimodal fusion in the classification of RE, integrating endoscopic images, clinical symptoms, esophageal pH monitoring, etc.

## Figures and Tables

**Figure 1:** The characteristic of the datasets.

**Figure 2:** The flowchart of the study.

**Figure 3:** Confusion matrix of the models.

**Figure 4:** Grad-CAM heatmap.

**Table 1:** Performance metrics of models and endoscopists.

	Models	Accuracy	Matthew's correlation coefficient	Cohen's kappa
*Validation dataset*				
	MobileNet	0.916	0.859	0.820
	ResNet	0.931	0.884	0.850
	Xception	0.938	0.896	0.860
	**EfficientNet**	**0.962**	**0.936**	**0.910**
	ViT	0.933	0.888	0.850
	ConvMixer	0.950	0.916	0.890

*Test dataset*				
	MobileNet	0.916	0.821	0.780
	ResNet	0.933	0.846	0.810
	Xception	0.936	0.852	0.810
	**EfficientNet**	**0.957**	**0.884**	**0.850**
	ViT	0.938	0.854	0.820
	ConvMixer	0.943	0.861	0.820
	Junior endoscopist	*0.916*	*0.820*	*0.780*
	Senior endoscopist	*0.945*	*0.864*	*0.830*

The bold figures indicate the highest numeric values.

## Data Availability

The dataset used to support the findings of the study is from HyperKvasir, which is now the largest open dataset of the gastrointestinal endoscopy (https://datasets.simula.no/hyper-kvasir/).
